This article has been retracted.

# Influence of Personalized Health Management Model Based on Internet Mode on Self-Management Ability and Life Quality of Patients with Chronic Diseases Undergoing Physical Examination

**DOI:** 10.1155/2022/4434436

**Published:** 2022-08-09

**Authors:** Li Qiao, Ruijuan Li

**Affiliations:** ^1^Physical Examination Department, Yuncheng First Hospital Yuncheng, Shanxi 044000, China; ^2^The Pain Department, Yuncheng First Hospital Yuncheng, Shanxi 044000, China

## Abstract

**Objective:**

To explore the influence of personalized health management model based on the Internet mode on self-management ability and life quality of patients with chronic diseases of physical examination.

**Methods:**

Sixty patients with chronic diseases who went through physical examination from February 2019 to April 2021 were enrolled in our hospital. The patients were arbitrarily assigned into control and research group. The former group received routine nursing, and the latter group received personalized health management mode based on the Internet mode. The nursing satisfaction, self-management behavior ability, blood pressure level, physiological index, mastery of health knowledge, and life quality scores were compared.

**Results:**

In terms of nursing satisfaction, the research group was very satisfied in 20 cases, satisfactory in 9 cases, and general in 1 case, with a satisfaction rate of 100.00%; In the control group, 15 cases were very satisfied, 9 cases were satisfied, 1 case was general, 5 cases were not satisfied, and the satisfaction rate was 83.33%; The nursing satisfaction of the research group was higher (*P* < 0.05). Compared with the self-management behavior ability, the scores of diet control, regular medication, correct medication, and smoking cessation in the research group were remarkably higher (*P* < 0.05). There exhibited no significant difference in blood pressure level before intervention (*P* > 0.05); after intervention, the blood pressure levels lessened. Compared with the control group, the systolic blood pressure and diastolic blood pressure of the research group were lower (*P* < 0.05). The levels of triglyceride, total cholesterol, low-density lipoprotein, and fasting blood glucose in the research group were remarkably lower (*P* < 0.05). Compared with the control group, the scores of health knowledge in the research group were remarkably higher, including the harm of smoking, the use of drugs, the importance of persisting in taking drugs, the pathogenesis of chronic diseases, the effect of emotional management on the disease, and the dietary awareness in the research group (*P* < 0.05). There exhibited no significant difference in the score of life quality before nursing (*P* > 0.05); after nursing, the score of life quality lessened, and the scores of physiological function, psychological function, social function, and health self-cognition in the research group were lower (*P* < 0.05).

**Conclusion:**

The personalized health management model based on the Internet mode can effectively enhance the chronic disease physiological indexes such as blood pressure, blood lipids, and blood sugar and improve the self-management ability of the patients with chronic disease, which is worth further popularizing and applying in the clinical physical examination in clinic.

## 1. Introduction

At present, the aging of the social population is accelerating, the incidence and prevalence of chronic diseases in the elderly are high, and the number of patients with diabetes, hypertension, and Alzheimer's disease is increasing day by day, which brings a heavy burden to the society and families [1]. The reality of the aging population requires us to develop effective and sustainable interventions to solve the problems of prevention and management of chronic diseases in the elderly. One of the main tasks of the current management process of prevention and treatment of chronic diseases in the elderly in China is follow-up management [1, 2]. The main forms of follow-up include community follow-up provided by community hospitals and remote follow-up (such as telephone follow-up) and family follow-up provided by general hospitals. However, in the current community hospital follow-up due to weak community medical strength, there are insufficient coverage, poor follow-up effect, low patient acceptance, and other shortcomings [2]. In the initial stage, chronic disease management in the community, more time invested by doctors, and health education forums have become a generally accepted way for the elderly with chronic diseases. However, the number of personnel with specialized professional qualifications is very rare. The professional quality of community general practitioners is generally low, unable to achieve accurate assessment and individual services for elderly chronic diseases. In the meantime, the elderly people's awareness and basic knowledge of early disease identification, diagnosis, and prevention are not enough, so it is necessary to strengthen the training and promotion of health literacy in this area. Take people with senile dementia, a special group of chronic diseases in the elderly, as an example. At present, the number of people with dementia is about 10 million, but the current medical situation of dementia in China is that “the consultation rate is very low.” The reasons are as follows: (1) the public's general understanding of the disease is not enough, such as that “dementia” is similar to “senile forgetfulness and senile confusion”; (2) doctors in community and grass-roots hospitals still lack specialized knowledge of cognitive disorders and effective diagnostic tools; (3) the congenital deficiency of the traditional mode of seeking medical treatment. The traditional mode of “queuing registration-nurse triage-specialist treatment-medicine collection-follow-up observation-revisit” is extremely tedious, which is also the reason for the low consultation rate of this kind of disease. Therefore, the promotion of scientific and intelligent health management and health literacy services is expected to enhance the physical and mental health and good life quality of the elderly. For example, moving the health management of the elderly so that they can enjoy health information services at home, in personalized management, timely communication with health care personnel, and reducing the waste of medical resources as well as providing medical data support for specific disease areas are beneficial [3].

In recent years, with the progress of medical technology and the extension of life expectancy, the global aging trend is also deepening, and chronic disease has increasingly become an important public health problem endangering people's health [4]. Chronic disease, that is, chronic noncommunicable disease (NCD), refers to a group of diseases represented by cardiovascular disease, malignant tumor, metabolic disease, and chronic obstructive pulmonary disease [5]. In particular, cardiovascular and metabolic chronic diseases, such as hypertension, hyperlipidemia, and diabetes, are not only related to genetic factors, but also related to patients' bad lifestyle, behavior habits, and high-salt, high-sugar, and high-fat diet [6]. If we can intervene in the early stage of the disease or when the body is in a state of subhealth and improve the bad lifestyle, it can greatly reduce the occurrence and development of chronic disease. Based on the Internet +'s health literacy model for elderly chronic diseases, it can include patients' registration on the intelligent APP interface, filling in basic health data sheets, self-health assessment, GPS positioning, establishment of electronic health files, data extraction, analysis, and statistics [7]. Some APP models can also learn from some experience but need to be localized and enhanced to suit the practical application of our population. Physical examination, as one of the means to detect abnormalities in the early stage, has been unable to meet the growing health needs of the people. With the enhancement of public awareness of health care, health management came into being. With the widespread popularity of the Internet and big data, the development of online remote health management model is in full swing; intelligent, information-based, personalized medical data management is the general trend [8]. The exploration of the management model of cardiovascular and metabolic chronic diseases has been very mature, but most of them focus on the chronic patients who have obvious adverse symptoms, hospital treatment, and community management. The research on the subhealth population found by physical examination is less [9, 10]. In this study, we carried out a personalized health management model based on the Internet model for people with abnormal blood pressure, blood lipids, and blood sugar found by physical examination and observed the effect of this model on the life quality and self-management ability.

## 2. Patients and Methods

### 2.1. Normal Information

Sixty patients with chronic diseases who went through physical examination from February 2019 to April 2021 were enrolled in our hospital. The patients were arbitrarily assigned into control and research group. In the former group, the age ranged from 18 to 74 years old, with an average of 38.43 ± 4.53 years, including 18 males and 12 females; in the latter group, the age ranged from 18 to 76 years old, with an average of 38.67 ± 4.58 years, including 16 males and 14 females. There exhibited no statistical significance in the general data (*P* > 0.05). This study was permitted by the Medical Ethics Association of our hospital, and all patients noticed informed consent.

Inclusion criteria are as follows: (1) during the study period, the indexes of blood pressure, blood lipid, and fasting blood glucose exceeded the normal range. According to the relevant guidelines and laboratory testing instruments, the diagnostic criteria were set as follows [11]: systolic blood pressure ≥140 mmHg (1 mmHg =0.133 kPa) and/or diastolic blood pressure ≥90 mmHg, triglyceride >1.7 mmol/L, total cholesterol >5.18 mmol/L, low-density lipoprotein >3.12 mmol/L, and fasting blood glucose >6.1 mmol/L; (2) patients with clear consciousness and normal reading ability; (3) proficient in the use of mobile phone, WeChat.

Exclusion criteria are as follows: (1) patients with severe cardiovascular and cerebrovascular diseases in the past; (2) patients with other chronic diseases or malignant tumors such as hepatitis, tuberculosis, and renal insufficiency; (3) abnormal and critical values found in the department's “Revised Management of Important Abnormal Results” system during the examination and need to notify the medical examiners who visit the abnormal specialist; (4) the examiners who cannot accept investigation and research due to other diseases.

### 2.2. Treatment Methods

#### 2.2.1. Control Group

Routine health visit management was adopted in the department; that is, at 1, 3, and 6 months after the examination, the return visitors made a telephone health visit to the physical examiners to understand their recent blood pressure, blood lipids, and blood sugar control; give health advice on diet, exercise, monitoring, and drug treatment; and reply and record the health problems consulted by the physical examiners as soon as possible.

#### 2.2.2. Research Group

Implement the personalized health management model based on the Internet model. (1) Set up a personalized health management team: set up four teams, each with fixed doctors, nurses, and health managers, as well as mobile dietitians, rehabilitation therapists, psychological counselors, and Internet assistant managers. The group formulates the job responsibilities, and each member performs his or her own duties and gives full play to his or her professional advantages. According to the sequence of physical examination, 30 subjects in the experimental group were assigned into three management teams, 10 cases in each group, which were managed by group mode. The group type is not only a group formed by professional health managers such as doctors and nurses, but also a group formed by the physical examiners themselves; in the meantime, the two sides jointly form a “manage-be managed” group; (2) establish personalized health examination files: set up personalized health examination files for those who are enrolled in the research group, fill in the health examination questionnaire during the examination, and have an in-depth understanding of the information of each examiner, including general information, such as marital status, education level, type of medical insurance, past history, current medical history, and family history; smoking, drinking, diet, exercise, sleep, and other living conditions as well as personal psychological factors. Doctors effectively analyze the health files of physical examiners, comprehensively evaluate their physical and mental status, find out the existing or potential pathogenic factors, analyze the causes, formulate personalized management plans, and then implement health intervention; (3) make full use of the Internet intelligent means: the WeChat official account service module of Health Management Section includes physical examination appointment, report inquiry, health questionnaire, and other items and uploads popular science articles regularly. Physical examiners follow the official WeChat account, upload self-tested health data using the Internet, and conduct targeted health return visits after team members' analysis. The adoption of the Internet +'s information intelligent health management method can make the physical examination more convenient and faster and free from the multiple restrictions of time, space, and place; (4) personalized health management intervention: (a) determine the time of health management intervention and formulate the intervention plan. The time is 6 months, once a month, according to the chronic disease index records fed back by the physical examiners; health return visits are carried out by means of phone calls, text messages, WeChat, etc., and door-to-door health education guidance is also available depending on the situation; (b) advocating peer education and allowing family members of physical examiners to participate in health management can, to a certain extent, encourage physical examiners and couples to supervise each other and improve their self-management ability and behavior together; (c) regular monitoring of indicators guide people who are assisted in physical examination to use chronic disease health kit, including index monitoring time and record table, popular science publicity manual, sphygmomanometer, blood glucose meter, and weekly metering kit. Guide the correct use of the instrument, the matters needing attention in monitoring, and inform the importance of regular records; (d) diet and exercise management: there are dietitians and rehabilitation therapists in the management group to formulate diet and exercise prescriptions according to the past diet, exercise habits, and preferences of the physical examination. Dietitians and doctors cooperate with each other to design improvement methods according to local conditions in view of the current diet problems of physical examiners, such as those who eat faster, guide, and prolong the eating time. The diet should be light; control the intake of high-salt, high-fat, and high-sugar food; eat more fruits and vegetables; change bad eating habits; and correct unreasonable diet. Rehabilitation therapists make daily exercise plans, strengthen aerobic exercise, appropriately increase resistance training when the physical examiner's intensity load is satisfied, and guide the correct shape and posture; (e) regular and healthy lifestyle: guide the physical examiner to pay attention to the combination of work and rest in daily life, develop good living habits, maintain emotional stability, mental happiness, and ensure adequate sleep every day. And carry out health education on the harm of tobacco and alcohol, guide the physical examination to give up smoking and limit alcohol, pay attention to it step by step, and avoid withdrawal symptoms. The members of the management team should pay attention to communication during the return visit so as to appease the bad mood of the physical examination. Psychological counselors give lectures on mental health every month to relieve the psychological pressure of medical examiners on disease treatment; (5) adjust the personalized health management plan at any time: the doctors in the health management group adjust the personalized health management plan according to the content information fed back by the physical examiner's phone or WeChat and the chronic disease index uploaded by the Internet.

### 2.3. Observation Index

#### 2.3.1. Satisfaction

After consulting the literature and experts' discussion, we designed patients' follow-up satisfaction, a total of 10 items, and recorded patients' satisfaction with follow-up management mode, health education, medical and nursing service, and appointment registration process [12]. It is assigned into four dimensions: very satisfied, satisfied, general, and dissatisfied. Satisfaction rate = very satisfaction rate + satisfaction rate + general rate.

#### 2.3.2. Self-Management Behavior Ability

After the intervention, the self-management behavior ability questionnaire [13] was used to accurately evaluate the patients' self-management behavior ability: diet control, regular medication, correct medication, smoking cessation behavior. The results of the survey were expressed by scores, with a full score of 100. The higher the score, the stronger the patient's ability of self-management behavior.

#### 2.3.3. Blood Pressure Level

Before and after intervention, the levels of diastolic blood pressure and systolic blood pressure were recorded before and after intervention.

#### 2.3.4. Physiological Index

After intervention, the indexes of triglyceride, total cholesterol, low-density lipoprotein, and fasting blood glucose were recorded.

#### 2.3.5. Health Knowledge Questionnaire

Before and after intervention, the health knowledge questionnaire was adopted to evaluate the health knowledge mastery after intervention in different ways [14]. The main contents of the assessment are as follows: the harm of smoking, the use of drugs, the importance of insisting on taking drugs, the pathogenesis of chronic diseases, the influence of emotional management on the condition, and the dietary precautions. The highest score is 100, and the higher the score, the higher the patients' mastery of health knowledge.

#### 2.3.6. Life Quality Scale

Before and after intervention, the life quality scale consists of four subscales, including physical, psychological, social, and health self-awareness, with a total of 29 items [15]. The Cronbach's *α* coefficient of the scale is 0.79 to 0.91. The scale was scored by 1-5 grades. The lower the score, the higher the satisfaction.

### 2.4. Statistical Analysis

The data were processed by SPSS24.0 statistical software, and the measurement data were presented as ($\bar{x}\pm \text{s}$). Independent sample *t*-test was adpoted for intergroup comparison, and paired sample *t*-test was adopted for intragroup comparison. The counting data were expressed as a percentage and accepted the *χ*^2^ test. *P* < 0.05 indicates that the difference is statistically significant.

## 3. Results

### 3.1. Comparison of Nursing Satisfaction

In terms of nursing satisfaction, the research group was very satisfied in 20 cases, satisfactory in 9 cases, and general in 1 case, with a satisfaction rate of 100.00%; in the control group, 15 cases were very satisfied, 9 cases were satisfied, 1 case was general, and 5 cases were not satisfied, and the satisfaction rate was 83.33%; the nursing satisfaction of the research group was higher, and the difference between groups was statistically significant (*P* < 0.05). All the data results are indicated in Figure 1.

### 3.2. Comparison of Self-Management Behavior Ability

Regarding the self-management behavior ability, the scores of diet control, regular medication, correct medication, and smoking cessation in the research group were higher, and the difference between groups was statistically significant (*P* < 0.05). All the data results are indicated in Table 1.

### 3.3. Blood Pressure Level Comparison

There exhibited no significant difference in blood pressure level before intervention (*P* > 0.05); after intervention, the blood pressure levels lessened. Compared with the control group, the systolic blood pressure and diastolic blood pressure of the research group were lower, and the difference between groups was statistically significant(*P* < 0.05). All the data results are indicated in Table 2.

### 3.4. Comparison of Physiological Indexes

The levels of triglyceride, total cholesterol, low-density lipoprotein, and fasting blood glucose in the research group were remarkably lower, and the difference between groups was statistically significant (*P* < 0.05). All the data results are indicated in Table 3.

### 3.5. Comparison of Mastery of Health Knowledge

Compared with the control group, the scores of the harm of smoking, the way of drug use, the importance of persisting taking drugs, the pathogenesis of chronic diseases, and the influence of emotional management and dietary attention in the research group were higher, and the difference between groups was statistically significant (*P* < 0.05). All the data results are indicated in Figure 2.

### 3.6. Comparison of Life Quality Scores

There exhibited no significant difference in the score of life quality before nursing (*P* > 0.05); after nursing, the score of life quality lessened. Compared between the two groups, the scores of physiological function, psychological function, social function, and health self-cognition in the research group were lower, and the difference between groups was statistically significant (*P* < 0.05). All the data results are indicated in Table 4.

## 4. Discussion

With the improvement of people's living standards and the enhancement of health care awareness, more people begin to pay attention to the new field of health management [15]. The incidence of chronic diseases caused by global aging is increasing, which brings great impact and burden on individuals, families, and society. How to maximize the benefits of physical examination, enhance health management, and then achieve national health promotion is the eternal theme of the health industry [16]. NCD is a kind of disease with hidden onset, long incubation period, long and slow course of disease, persistent disease, lack of exact evidence of biological etiology, and no clear indication of “cure” [17]. The common chronic diseases are mainly cardio-cerebrovascular diseases, diabetes, malignant tumors, and chronic obstructive pulmonary diseases. It is predicted that by 2030, the total number of global chronic disease-related deaths will rise to 70% of the world's total deaths [18]. With the aggravation of the aging population in our country, the number of patients with chronic disease is increasing rapidly. The number of deaths caused by chronic disease has accounted for 85% of the total deaths in our country, and its disease burden has accounted for 70% of the total disease burden in our country [19]. Clinically, chronic diseases have a high incidence, which can have a great impact on human physical and mental health [20]. At present, it has been reported that taking targeted measures for the risk factors of chronic diseases and effective prevention and control can reduce the risk of chronic diseases and enhance their life quality [21]. As early as 2003, the World Health Organization report stressed that doctors can not only rely on doctors to promote the compliance of most patients with chronic diseases, doctors do not have enough time for individual intervention, and health education can effectively change patients' knowledge and behavior. It can effectively enhance the self-management ability of patients with chronic diseases and enhance their compliance. Chronic disease self-management (CDSM) is a modern biopsychosocial medical management model, which means that patients and their families undertake disease prevention and treatment activities consciously and actively with the assistance of medical staff [22]. The traditional collectivization and irregular health education model has been unable to meet the growing health needs of patients with chronic diseases, and individualized health education programs are in line with the development trend. Some countries have successfully applied this management model to the rehabilitation of various chronic diseases. In the process of health education, we can not only enhance the relationship between nurses and patients, but also obtain more disease knowledge, guide patients to change their bad behavior, and master the skills of disease self-monitoring and management through health education [23, 24]. Individualized health education is a kind of health education, which advocates to formulate individual clinical treatment and nursing programs for patients based on the actual clinical symptoms and disease characteristics of patients, so as to enhance the pertinence of disease prevention and treatment. It has important practical value to promote patients' awareness and level of self-care [25].

As an important part of clinical nursing work, health education plays a vital role in the recovery of patients' condition [26]. The study found that, combined with the pathological characteristics of chronic diseases and the condition of patients, the formulation of the best individual health education program can stimulate patients' attention to their own health, enhance their mastery of health knowledge, and establish a kind of clinical thinking [27]. In the meantime, it can also enhance patient compliance so as to promote the effect of standardized treatment, bring patients confidence in the treatment of diseases, and form a virtuous circle with each other. Patients can dynamically grasp their own health status; reduce the number of acute attacks of the disease; reduce the incidence, hospitalization rate, and hospitalization days; alleviate family medical expenses and reduce their economic pressure; and reduce the social medical burden. In addition, it is also reported that, compared with traditional health education, individualized health education has more practical significance in chronic diseases, such as the following: (1) it can improve patients' ability of self-management behavior; (2) it can enhance the stability of patients' mentality; (3) conducive to the development of patients' good eating habits; (4) patients' sense of self-worth has been improved; and (5) improve the life quality of patients [28–31]. The results indicated that the scores of health knowledge questionnaire and self-management behavior ability in the research group were remarkably higher, and the satisfaction rate of patients in the research group was also remarkably higher. It also shows that individual health education is more suitable for the management and recovery of patients with chronic diseases than traditional health education. After intervention, the physiological indexes of the research group were remarkably lower. This study adopts the personalized health management model based on the Internet mode, which brings together doctors and nurses with their own expertise, and each member gives full play to their own professional advantages and realizes the complementary disciplines. It can carry out omnidirectional and targeted health management for physical examiners [32, 33]. Professional sports rehabilitation experts and health managers formulate exercise prescriptions according to the personal situation of physical examiners; adopt scientific, planned, and reasonable exercise; increase body energy consumption; and gradually control body weight. Combined with the past eating habits of the physical examiners, the dieticians individualized the diet plan in line with the regional dietary characteristics, improved the dietary structure, and controlled the intake of sugar, salt, and lipids under the condition of ensuring the balanced nutrition of the physical examiners, so as to achieve the purpose of reducing fat and weight [34]. With the control of weight, the health problems caused by obesity also improved to a certain extent, and the blood pressure, blood lipids, and fasting blood glucose indexes of chronic patients also lessened. The personalized health management model based on the Internet mode makes full use of the development and application of information in health management; breaks through the restrictions of time, space, and place; and transmits the information and data uploaded through the Internet to medical staff in real time. Medical staff timely feedback, to a certain extent, also played a role in prompting and supervising the physical examination [35–37]. After health intervention, the scores of self-management ability were enhanced, because the score of self-management ability was self-evaluation of physical examiners, and the subjective factors had great influence, so the score after intervention was more practical. After the research group adopted the mode of personalized health management based on the Internet mode, the score of self-management ability of physical examiners was remarkably higher. Considering the psychological impact of chronic illness on patients, we invite psychological counselors to popularize relevant knowledge to make them understand the importance of self-management, enhance their enthusiasm for participation, and then promote their self-management ability. With the improvement of the self-management ability of the physical examiners, the control over an increase of good lifestyle and the clinical-related physiological indicators are also better controlled. The results were consistent with the results of Chen Dan and Liu Shengxiang [38, 39]. After the group health management of stroke patients, the scores of self-management behavior and life quality were enhanced, and the clinical indexes were also promoted. This study advocates peer education, fully considers the importance of the role of family members, encourages family members to participate, and takes the physical examiner as the main body and the family as the center. The physical examiner feels the care and attention of the family members, which not only enhances the confidence in overcoming the disease, but also helps to improve the ability of self-management and promote the rehabilitation of the disease [40, 41]. Personalized health management takes full account of the personal living habits and characteristics of physical examiners, which can reduce their rebellious psychology caused by behavior restrictions, enhance their bad mood, be more easily accepted by physical examiners, improve their spirit of ownership, and increase their own participation [42–44].Our study still has some shortcomings. Firstly, the quality of this study is limited due to the small sample size we included in the study. Secondly, this research is a single-center study, and our findings are subject to some degree of bias. Therefore, our results may differ from those of large-scale multicenter studies from other academic institutes. Our research is still clinically significant, and further in-depth investigations will be carried out in the future. The same idea can be found in the study put forward by Bian [45]. They have applied new methods in the study, and the conclusions drawn can also give some support to this study.

In summary, the personalized health management model based on the Internet mode can effectively enhance the chronic disease physiological indexes such as blood pressure, blood lipids, and blood sugar and improve the self-management ability of the patients with chronic diseases. It is worth further popularizing and applying in clinical physical examination in clinic.

## Figures and Tables

**Figure 1:** Comparison of nursing satisfaction between the two groups.

**Figure 2:** Comparison of mastery of health knowledge between the two groups.

**Table 1:** Comparison of self-management behavior ability between the two groups [$\bar{x}\pm \text{s}$, points].

Grouping	*N*	Control diet	Take medicine regularly	Correct use of drugs	Quitting smoking behavior
Control group	30	15.33 ± 3.11	14.59 ± 2.13	14.33 ± 2.34	14.66 ± 1.34
Research group	30	21.14 ± 1.22	20.69 ± 1.25	21.93 ± 0.53	20.81 ± 1.21
*t*		9.525	13.528	17.349	18.657
*P*		<0.05	<0.05	<0.05	<0.05

**Table 2:** Comparison of blood pressure between the two groups [$\bar{x}\pm \text{s}$].

Grouping	*N*	Systolic blood pressure (mmHg)		Diastolic pressure (mmHg)	
		Before intervention	After intervention	Before intervention	After intervention
Control group	30	151.38 ± 12.64	143.14 ± 8.31	100.94 ± 13.52	94.68 ± 3.56
Research group	30	151.59 ± 12.45	134.69 ± 7.34	100.91 ± 13.35	89.31 ± 5.23
*t*		0.064	4.174	0.008	4.649
*P*		>0.05	<0.05	>0.05	<0.05

**Table 3:** Comparison of physiological indexes between the two groups [$\bar{x}\pm \text{s}$, mmol/L].

Grouping	*N*	Triacylglycerol	Total cholesterol	Low density lipoprotein	Fasting blood glucose
Control group	30	3.41 ± 0.75	6.09 ± 0.66	3.75 ± 0.94	8.32 ± 0.75
Research group	30	2.15 ± 0.42	5.23 ± 0.43	3.15 ± 0.65	7.24 ± 0.86
*t*		8.028	5.979	2.875	5.183
*P*		<0.05	<0.05	<0.05	<0.05

**Table 4:** Comparison of life quality scores between the two groups [$\bar{x}\pm \text{s}$, points].

Grouping	*N*	Physiological function		Psychological function		Social function		Healthy self-cognition	
		Before nursing	After nursing	Before nursing	After nursing	Before nursing	After nursing	Before nursing	After nursing
Control group	30	15.65 ± 4.51	13.95 ± 2.67^a^	16.78 ± 3.96	14.89 ± 4.55^a^	18.53 ± 3.76	16.37 ± 2.42^a^	15.58 ± 3.55	13.78 ± 1.53^a^
Research group	30	15.67 ± 4.52	11.82 ± 2.56^b^	16.76 ± 3.78	12.77 ± 1.53^b^	18.57 ± 3.53	12.64 ± 3.67^b^	15.53 ± 3.75	10.85 ± 2.42^b^
*t*		0.017	3.53	0.020	2.418	0.042	4.647	0.053	5.605
*P*		>0.05	<0.05	>0.05	<0.05	>0.05	<0.05	>0.05	<0.05

Note: Comparison before and after nursing in the control group, ^a^*P* < 0.05; comparison before and after nursing in the research group, ^b^*P* < 0.05.

## Data Availability

The datasets used and analyzed during the current study are available from the corresponding author upon reasonable request.
